# Grey relational analysis method for typhoon vulnerability assessment of civil engineering structures based on the 2-tuple linguistic neutrosophic number

**DOI:** 10.1371/journal.pone.0277539

**Published:** 2022-11-15

**Authors:** Yong Qi, Chen Zhu, Fang Wang, Yu Xia

**Affiliations:** 1 College of Environment and Civil Engineering, Chengdu University of Technology, Chengdu, Sichuan, China; 2 State Key Laboratory of Geohazard Prevention and Geoenvironment Protection, Chengdu, Sichuan, China; 3 China Craftsmen International Engineering Design Co., Ltd., Chengdu, Sichuan, China; Hefei University of Technology, CHINA

## Abstract

As one of the severe natural disasters, typhoon hazard brings tremendous tragedy to human beings. The foreland in the southeast of China is one of the most typhoon prone areas in the world. There are amount of damage of civil engineering structures induced by typhoon every year. Especially for the spacious villages, the low-rise buildings are vulnerable to typhoon so that many of them are destroyed regionally. The typhoon vulnerability assessment of civil engineering structures is a classical multiple attribute group decision making (MAGDM) issues. In this paper, the 2-tuple linguistic neutrosophic number grey relational analysis (2TLNN-GRA) method is built based on the grey relational analysis (GRA) and 2-tuple linguistic neutrosophic sets (2TLNSs) with incomplete weight information. For deriving the weight information of the attribute, an optimization model is built on the basis of the GRA, by which the attribute weights can be decided. Then, the optimal alternative is chosen through calculating largest relative relational degree from the 2-tuple linguistic neutrosophic number positive ideal solution (2TLNNPIS) which considers both the largest grey relational coefficient (GRC) from the 2TLNNPIS and the smallest GRC form 2-tuple linguistic neutrosophic number negative ideal solution (2TLNN NIS). Then, combine the traditional fuzzy GRA model with 2TLNNSs information, the 2TLNN-GRA method is established and the computing steps for MAGDM are built. Finally, a numerical example for typhoon vulnerability assessment of civil engineering structures has been given and some comparisons is used to illustrate advantages of 2TLNN-GRA method.

## 1. Introduction

The multiple attribute group decision-making (MAGDM) refers to integrating and ranking the criterion values of multiple schemes under multiple criteria [1–3]. Due to the complexity of the decision-making environment and the limited cognition of decision-makers, it is difficult for decision-makers to give accurate evaluation information in actual decision-making [4–7]. In 1986, Atanassov [8] defined the intuitionistic fuzzy sets (IFSs) on the fuzzy theory proposed by Zadeh [9], adding the degree of non-membership and hesitation to describe the degree of uncertainty of "one or the other", which can be more delicate than fuzzy sets. Smarandache [10] put forward the concept of neutrosophic sets (NSs) in 1999, which can clearly quantify uncertain and inconsistent information, and reflect the dynamic information of things, phenomena or ideas. The NSs add an independent uncertainty measure, which is an extension and generalization of fuzzy sets. Wang et al. [11] defined the 2TLNSs which all decision values are expressed by 2-tuple linguistic term sets (2TLs).

There are three shortcomings in disposing of the MAGDM problems under 2TLNSs environment that to form our incentives in the following:

1. The existing decision methods just consider distance-based similarity degree [12]. How to investigate the decision methods consider the shape-based similarity degree. is an interesting and hot topic. For this reason, the first incentive of this paper is to build the new shape-based similarity degree decision methods.
2. The existing weight determining methods just consider completely known weight information [13, 14]. How to investigate the weight determining method consider incompletely known weight information is an interesting and hot topic. For this reason, the second third incentive of this paper is to build new weight determining method, which can deal with incompletely known weight information.
3. The concept of vulnerability was first proposed in the military field to describe the vulnerability of an aircraft or ship’s hull to physical collisions. It was not until 1968 that the concept of structural fragility was first proposed in the Ronan Point apartment collapse to express the ability of a structure to withstand disproportionate collapse. Therefore, it is urgent for researchers in related disciplines to conduct exploratory research in this field to enrich the research content of typhoon disasters in Chinese. The typhoon disaster assessment of civil engineering structures in Chinese is still in a blank state. Therefore, it is urgent for researchers in related disciplines to conduct exploratory research in this field to enrich the research content of typhoon disasters in my country. The typhoon vulnerability assessment study of civil engineering structures has two meanings: (a) according to the typhoon disaster prediction, designers can improve the structure’s typhoon resistance ability according to the different typhoon vulnerability of the structure; (b) according to the typhoon disaster Loss assessment research, decision-making departments can provide a basis for government and enterprise typhoon disaster loss estimates. The typhoon vulnerability assessment of civil engineering structures is a classical MAGDM issues. Thus, the third incentive of this paper is to build new decision methods for typhoon vulnerability assessment of civil engineering structures.

On this basis, combined with the characteristics of typhoon vulnerability assessment of civil engineering structures, a new MAGDM method for typhoon vulnerability assessment of civil engineering structures in 2TLNSs environment is proposed. Specific research points are listed as follows:

1. In this paper, the 2-tuple linguistic neutrosophic number grey relational analysis (2TLNN-GRA) method is built based on the GRA and 2TLNSs with incomplete weight information. The 2TLNN-GRA investigate the decision methods consider the shape-based similarity degree.
2. For deriving the incompletely known weight information of the attribute, an optimization model is built on the basis of the 2TLNN-GRA, by which the attribute weights can be decided. Then, the optimal alternative is chosen through calculating largest relative relational degree from the 2-tuple linguistic neutrosophic number positive ideal solution (2TLNNPIS) which considers both the largest grey relational coefficient (GRC) from the 2TLNNPIS and the smallest GRC form 2-tuple linguistic neutrosophic number negative ideal solution (2TLNN NIS). Then, combine the traditional fuzzy GRA model with 2TLNNSs information, the 2TLNN-GRA method is established and the computing steps for MAGDM are built.
3. Finally, a numerical example for typhoon vulnerability assessment of civil engineering structures has been given and some comparisons is used to illustrate advantages of 2TLNN-GRA method. This paper mainly provides method guidance and technical support for the realization of typhoon damage assessment and prediction of low-rise building structures in the southeastern coastal villages and towns of my country through the preliminary research on the typhoon vulnerability assessment of civil engineering structures. This has far-reaching significance for the decision-making of typhoon prevention and disaster mitigation in the public sector, infrastructure construction in villages and towns, and even national security and stability.

In order to do so, the reminder structure of such built paper proceeds. The related literature review is introduced in Sec. 2. The 2TLNNSs is introduced in Sec. 3. The 2TLNN-GRA method is built for MAGDM in Sec. 4. A numerical example for typhoon vulnerability assessment of civil engineering structures is given and some comparisons are also done in Sec. 5. Sec. 6 gives some the conclusions.

## 2. Related literature review

Due to the complexity of the decision-making environment and the limited cognition of decision-makers, it is difficult for decision-makers to give accurate evaluation information in actual decision-making. In this case, how to effectively solve the above problems and make more reasonable decisions, the research on relevant decision-making methods is particularly important. In 1986, Atanassov [8] expanded on the fuzzy theory proposed by Zadeh [9], adding the degree of non-membership and hesitation to describe the degree of uncertainty of "one or the other", which can be more delicate than fuzzy sets. Therefore, it is more flexible and applicable than fuzzy sets, and has been widely used in many fields such as economy, management, engineering design, etc., especially in the field of soft decision-making. Xu [15] studied a class of MADM problems in which the attribute value is intuitionistic fuzzy sets (IFSs) and the decision maker has a preference for the scheme, defined a series of judgment matrices, and used the linear programming model to determine the weight of the attribute. Xia and Xu [16] established a similarity measurement method of IFSs for MADM. Szmidt and Kacprzyk [17] proposed IFSs kernels and consistency criteria for imprecise information decision-making. Liao et al. [18] aimed at the problem of information loss caused by eliminating expert opinions in MAGDM methods and the combination of MAGDM and IFSs. Khaleie and Fasanghari [19] used intuitionistic fuzzy entropy to comprehensively consider subjective and objective factors and calculate the weight of experts. Gu et al. [20] proposed an intuitionistic fuzzy MADM scheme optimization method based on correlated information and prospect theory. Pei et al. [21] studied the group decision-making problem with low consensus characteristics based on the intuitionistic fuzzy theory. Ren, Gao and Yang [22] used IFSs information and construct fuzzy decision-making models based on regret theory. Smarandache [10] put forward the neutrosophic sets (NSs) in 1999. The NSs describes the relationship between the event and the fuzzy concept represented by the membership degree of the element and the set. Each element of it contains the true membership function, the uncertain membership function and the distortion membership function. The NSs add an independent uncertainty measure, which is an extension and generalization of fuzzy sets. Since the theory of NSs was put forward, it has been widely used in many fields such as social problems [23], artificial intelligence and control systems [24, 25], image processing, medical diagnosis [26], and enterprise management [27, 28]. Wang et al. [11] defined the 2TLNSs which all decision values are expressed by 2-tuple linguistic term sets (2TLs). Wu et al. [13] defined some new Hamy mean fused information operators along with 2TLNSs.

As a serious natural disaster, typhoon disaster has brought huge disasters to human beings. The southeastern coastal area of my country is one of the areas where typhoons land most frequently in the world. Affected by typhoons, a large number of civil engineering structures are damaged by wind disasters every year. Especially in the vast villages and towns, low-rise buildings have poor wind resistance and often regional damage collapse phenomenon. In order to evaluate and predict the typhoon disaster losses of civil engineering structures, so as to provide a basis for the decision-making of typhoon prevention and disaster reduction in the public sector. The concept of vulnerability was first proposed in the military field to describe the vulnerability of an aircraft or ship’s hull to physical collisions. It was not until 1968 that the concept of structural fragility was first proposed in the Ronan Point apartment collapse to express the ability of a structure to withstand disproportionate collapse. Successively, Lind [29] defined structural vulnerability based on probability as the ratio of the failure probability of a structurally damaged system to the failure probability of an undamaged system. While Lu et al. [30] defined the combination of components and possible failures of the structure. Wang et al. [31] studied the perceptions and personal experiences of some migrants living in Shanghai of typhoon hazards. Zhang et al. [32] developed a reliability-based vulnerability method for evaluating the typhoon induced wind risk of residential buildings in Japan. Morin et al. [33] studied the vulnerability to typhoon hazards for coastal informal settlements of Metro Manila. Nguyen et al. [34] analyzed the vulnerability of Vietnam to typhoons along with a spatial assessment on the basis of hazards, exposure and adaptive capacity. Guo et al. [35] coped with the vulnerability assessment issues for power transmission lines under typhoon weather on the basis of cascading failure state transition information diagram. Kim et al. [36] analyzed the typhoon vulnerability in South Korea through utilizing damage record model of typhoon Maemi. Ku et al. [37] solved the coastal vulnerability assessment issues of sea-level rise associated along with typhoon-induced surges in South Korea. Nguyen et al. [38] assessed the urban greenspace vulnerability to typhoon in Taiwan. Our country is still in a blank state in the field of typhoon disaster assessment of civil engineering structures. Therefore, it is urgent for researchers in related disciplines to conduct exploratory research in this field to enrich the research content of typhoon disasters in Chinese.

## 3. Preliminaries

### 3.1. 2-tuple linguistic term sets (2TLTSs)

Herrera and Martinez [39] defined the 2TLTSs.

Let *lδ* = {*ls*_*i*_ | *i* = 0,1,2,⋯, *M*} be the linguistic term sets (LTSs). Any label, *ls*_*i*_ represents a possible value through the given linguistic variable.

**Definition 1 [39]**. Let *β* be the fused result of labels assessed in the given *lδ*, i.e., the result of a symbolic fused operation, *β* ∈ [0, *M*], being *M* the cardinality of *lδ*. Let *i* = *round*(*β*) and *α* = *β* − *i* be two values, *i* ∈ [0, *M*] and *α* ∈ [−0.5, 0.5) then *α* is named the symbolic translation.

**Definition 2 [39]**. Let *lδ* = {*ls*_*i*_ | *i* = 0,1,2,⋯, *M*} be the LTSs and *β* ∈ [0, *M*] is the value representing the fused result of defined linguistic symbolic. Then the function Δ used to obtain the 2-tuple linguistic information equivalent to *β* is:

$$\Delta :\left[0,M\right]\to l\delta \times \left[-0.5,\left.0.5\right)\right.,$$ (1)

$$\Delta \left(\beta \right)=\left\{\begin{array}{l} ls_{i},\;i=round\left(\beta \right)\\ \alpha =\beta -i,\alpha \in \left[-0.5,\left.0.5\right)\right. \end{array}\right.,$$ (2)

where round(.) is the round operation, *ls*_*i*_ has the closest label to *β* and *α* is the symbolic translation value.

**Definition 3 [39]**. Let *lδ* = {*ls*_*i*_ | *i* = 0,1,2,⋯, *M*} be the LTSs and (*ls*_*i*_, *β*) be a 2-tuple. There is the function Δ^−1^, such that, from a 2-tuple (*ls*_*i*_, *β*) it returns the corresponding numerical value *β* ∈ [0, *M*] ⊂ *R*.


$$\Delta^{-1}:l\delta \times \left[-0.5,\left.0.5\right)\right.\to \left[0,M\right],$$ (3)

$$\Delta^{-1}\left(ls_{i},\beta \right)=i+\beta =\theta ,$$ (4)

### 3.2. Single-valued neutrosophic sets (SVNSs)

Let *X* be a fix set, the SVNSs *η* is depicted as [40]:

$$\eta =\left\{\left.\left(x,\phi_{\eta }\left(x\right),\varphi_{\eta }\left(x\right),\gamma_{\eta }\left(x\right)\right)\right|x\in X\right\}$$ (5)

where *ϕ*_*η*_(*x*), *φ*_*η*_(*x*), *γ*_*η*_(*x*) ∈ [0,1] represent the truth-membership, indeterminacy membership and falsity-membership, and meets the condition 0 ≤ *ϕ*_*η*_(*x*) + *φ*_*η*_(*x*) + *γ*_*η*_(*x*) ≤ 3.

### 3.3. 2TLNSs

Wang et al. [11] devised the 2TLNSs.

**Definition 4 [11]**. Let *lδ* = {*ls*_*i*_ | *i* = 0,1,2,⋯, *M*} be the LTSs. Any label *ls*_*i*_ depicts a possible linguistic information, and *lδ* = {*ls*_0_ = *exceedingly terrible*, *ls*_1_ = *very terrible*, *ls*_2_ = *terrible*, *ls*_3_ = *medium*, *ls*_4_ = *well*, *ls*_5_ = *very well*, *ls*_6_ = *exceedingly well*.}, then the 2TLNSs is described as:

$$l\delta =\langle \left(ls_{t},\alpha ,\right),\left(ls_{i},\beta \right),\left(ls_{f},\chi \right)\rangle$$ (6)

where Δ^−1^(*ls*_*t*_, *α*,), Δ^−1^(*ls*_*i*_, *β*), Δ^−1^(*ls*_*f*_, *χ*) ∈ [0, *M*] represent the truth-membership, indeterminacy-membership and the falsity-membership which are expressed by 2-tuple linguistic variables and meets the condition:

$$0\leq \Delta^{-1}\left(ls_{\alpha },\phi \right)+\Delta^{-1}\left(ls_{\beta },\varphi \right)+\Delta^{-1}\left(ls_{\chi },\gamma \right)\leq 3M$$ (7)

**Definition 5 [11]**. Let $l\delta_{1}=\langle \left(ls_{t_{1}},\alpha_{1},\right),\left(ls_{i_{1}},\beta_{1}\right),\left(ls_{f_{1}},\chi_{1}\right)\rangle$, $\delta_{2}=\langle \left(ls_{t_{2}},\alpha_{2},\right),\left(ls_{i_{2}},\beta_{2}\right),\left(ls_{f_{2}},\chi_{2}\right)\rangle$ be two 2TLNNs, the operation is defined:

1.
$l\delta_{1}⊕l\delta_{2}=\left\{\begin{array}{l} \Delta \left(M\left(\frac{\Delta^{-1}\left(ls_{t_{1}},\alpha_{1},\right)}{M}+\frac{\Delta^{-1}\left(ls_{t_{2}},\alpha_{2},\right)}{M}-\frac{\Delta^{-1}\left(ls_{t_{1}},\alpha_{1},\right)}{M}\cdot \frac{\Delta^{-1}\left(ls_{t_{2}},\alpha_{2},\right)}{M}\right)\right),\\ \Delta \left(M\left(\frac{\Delta^{-1}\left(ls_{i_{1}},\beta_{1}\right)}{M}\cdot \frac{\Delta^{-1}\left(ls_{i_{2}},\beta_{2}\right)}{M}\right)\right),\Delta \left(k\left(\frac{\Delta^{-1}\left(ls_{f_{1}},\chi_{1}\right)}{M}\cdot \frac{\Delta^{-1}\left(ls_{f_{1}},\chi_{1}\right)}{M}\right)\right) \end{array}\right\};$

2.
$l\delta_{1}⊗l\delta_{2}=\left\{\begin{array}{l} \Delta \left(M\left(\frac{\Delta^{-1}\left(ls_{t_{1}},\alpha_{1},\right)}{M}\cdot \frac{\Delta^{-1}\left(ls_{t_{2}},\alpha_{2},\right)}{M}\right)\right),\\ \Delta \left(M\left(\frac{\Delta^{-1}\left(ls_{i_{1}},\beta_{1}\right)}{M}+\frac{\Delta^{-1}\left(ls_{i_{2}},\beta_{2}\right)}{M}-\frac{\Delta^{-1}\left(ls_{i_{1}},\beta_{1}\right)}{M}\cdot \frac{\Delta^{-1}\left(ls_{i_{2}},\beta_{2}\right)}{M}\right)\right),\\ \Delta \left(M\left(\frac{\Delta^{-1}\left(ls_{f_{1}},\chi_{1}\right)}{M}+\frac{\Delta^{-1}\left(ls_{f_{2}},\chi_{2}\right)}{M}-\frac{\Delta^{-1}\left(ls_{f_{1}},\chi_{1}\right)}{M}\cdot \frac{\Delta^{-1}\left(ls_{f_{2}},\chi_{2}\right)}{M}\right)\right) \end{array}\right\};$

3.
$\lambda l\delta_{1}=\left\{\Delta \left(M\left(1-{\left(1-\frac{\Delta^{-1}\left(ls_{t_{1}},\alpha_{1},\right)}{M}\right)}^{\lambda }\right)\right),\Delta \left(M{\left(\frac{\Delta^{-1}\left(ls_{i_{1}},\beta_{1}\right)}{M}\right)}^{\lambda }\right),\Delta \left(M{\left(\frac{\Delta^{-1}\left(ls_{f_{1}},\chi_{1}\right)}{M}\right)}^{\lambda }\right)\right\},\lambda >0;$

4.
$l\delta_{\text{1}}^{\lambda }=\left\{\Delta \left(M{\left(\frac{\Delta^{-1}\left(ls_{t_{1}},\alpha_{1},\right)}{M}\right)}^{\lambda }\right),\Delta \left(M\left(1-{\left(1-\frac{\Delta^{-1}\left(ls_{i_{1}},\beta_{1}\right)}{M}\right)}^{\lambda }\right)\right),\Delta \left(M\left(1-{\left(1-\frac{\Delta^{-1}\left(ls_{f_{1}},\chi_{1}\right)}{M}\right)}^{\lambda }\right)\right)\right\},\lambda >0;$

According to Definition 2, the operation laws are defined.

1.
$l\delta_{1}⊕l\delta_{2}=l\delta_{2}⊕l\delta_{1},l\delta_{1}⊗l\delta_{2}=l\delta_{2}⊗l\delta_{1},{\left({\left(l\delta_{1}\right)}^{\lambda_{1}}\right)}^{\lambda_{2}}={\left(l\delta_{1}\right)}^{\lambda_{1}\lambda_{2}};$

2.
$\lambda \left(l\delta_{1}⊕l\delta_{2}\right)=\lambda l\delta_{1}⊕\lambda l\delta_{2},\;{\left(l\delta_{1}⊗l\delta_{2}\right)}^{\lambda }={\left(l\delta_{1}\right)}^{\lambda }⊗{\left(l\delta_{2}\right)}^{\lambda };$

3.
$\lambda_{1}l\delta_{1}⊕\lambda_{2}l\delta_{1}=\left(\lambda_{1}+\lambda_{2}\right)l\delta_{1},\;{\left(l\delta_{1}\right)}^{\lambda_{1}}⊗{\left(l\delta_{1}\right)}^{\lambda_{2}}={\left(l\delta_{1}\right)}^{\left(\lambda_{1}+\lambda_{2}\right)}.$

**Definition 6 [11]**. Let *lδ* = 〈(*ls*_*t*_, *α*,), (*ls*_*i*_, *β*), (*ls*_*f*_, *χ*)〉 be a 2TLNN, the score and accuracy functions of *lδ* is expressed:

$$s\left(l\delta \right)=\frac{\left(2M+\Delta^{-1}\left(ls_{t},\alpha ,\right)-\Delta^{-1}\left(ls_{i},\beta \right)-\Delta^{-1}\left(ls_{f},\chi \right)\right)}{3M},s\left(l\delta \right)\in \left[0,1\right]$$ (8)

$$h\left(l\delta \right)=\frac{1}{M}\left(\Delta^{-1}\left(ls_{t},\alpha ,\right)-\Delta^{-1}\left(ls_{f},\chi \right)\right),h\left(l\delta \right)\in \left[-1,1\right]$$ (9)

For *lδ*_1_ and *lδ*_2_, based on Definition 3, then

1.
$if\;s\left(l\delta_{1}\right)≺s\left(l\delta_{2}\right),\;then\;l\delta_{1}≺l\delta_{2};$

2.
$if\;s\left(l\delta_{1}\right)=s\left(l\delta_{2}\right),h\left(l\delta_{1}\right)≺h\left(l\delta_{2}\right),\;then\;l\delta_{1}≺l\delta_{2};$

3.
$if\;s\left(l\delta_{1}\right)=s\left(l\delta_{2}\right),h\left(l\delta_{1}\right)=h\left(l\delta_{2}\right),\;then\;l\delta_{1}=l\delta_{2}.$

### 3.4. The distance measurement of 2TLNNs

**Definition 7 [41]**. Let $l\delta_{1}=\langle \left(ls_{t_{1}},\alpha_{1},\right),\left(ls_{i_{1}},\beta_{1}\right),\left(ls_{f_{1}},\chi_{1}\right)\rangle$, $l\delta_{2}=\langle \left(ls_{t_{2}},\alpha_{2},\right),\left(ls_{i_{2}},\beta_{2}\right),\left(ls_{f_{2}},\chi_{2}\right)\rangle$, then the normalized Euclidean distance is:

$$ED\left(l\delta_{1},l\delta_{2}\right)=\sqrt{\frac{1}{3}\left(\begin{array}{l} {\left|\frac{\Delta^{-1}\left(ls_{t_{1}},\alpha_{1}\right)-\Delta^{-1}\left(ls_{t_{2}},\alpha_{2}\right)}{M}\right|}^{2}+{\left|\frac{\Delta^{-1}\left(ls_{i_{1}},\beta_{1}\right)-\Delta^{-1}\left(ls_{i_{2}},\beta_{2}\right)}{M}\right|}^{2}\\ +{\left|\frac{\Delta^{-1}\left(ls_{f_{1}},\chi_{1}\right)-\Delta^{-1}\left(ls_{f_{2}},\chi_{2}\right)}{M}\right|}^{2} \end{array}\right)}$$ (10)

### 3.5. The 2TLNNWG operators

**Definition 8 [11]**. Let $l\delta_{j}=\left\{\left(ls_{t_{j}},\alpha_{j}\right),\left(ls_{i_{j}},\beta_{j}\right),\left(ls_{f_{j}},\chi_{j}\right)\right\}\left(j=1,2,\ldots ,n\right)$ be a set of 2TLNNs, the 2TLNNWG operator is presented:

$$\begin{array}{l} \text{2TLNNWG}\left(l\delta_{1},l\delta_{2},\ldots ,l\delta_{n}\right)={\left(l\delta_{1}\right)}^{w_{1}}⊗{\left(l\delta_{2}\right)}^{w_{2}}\ldots ⊗{\left(l\delta_{n}\right)}^{w_{n}}=\overset{n}{\underset{j=1}{⊗}}{\left(l\delta_{j}\right)}^{w_{j}}\\ =\langle \begin{array}{l} \Delta \left(M\prod_{j=1}^{n}{\left(\frac{\Delta^{-1}\left(ls_{t_{j}},\alpha_{j}\right)}{M}\right)}^{w_{j}}\right),\Delta \left(M\left(1-\prod_{j=1}^{n}{\left(1-\frac{\Delta^{-1}\left(ls_{i_{j}},\beta_{j}\right)}{M}\right)}^{w_{j}}\right)\right),\\ \Delta \left(M\left(1-\prod_{j=1}^{n}{\left(1-\frac{\Delta^{-1}\left(ls_{f_{j}},\chi_{j}\right)}{M}\right)}^{w_{j}}\right)\right). \end{array}\rangle \end{array}$$ (11)

where *w*_*j*_ is weight of *lδ*_*j*_, which meets $0\leq w_{j}\leq 1,\sum_{j=1}^{n}w_{j}=1$.

## 4. GRA method for MAGDM issue with 2TLNNs

In this section, the 2TLNN-GRA method is defined for MAGDM. Suppose there are *m* defined decision alternatives {*ϕ*_1_, *ϕ*_2_, …*ϕ*_*m*_}, *n* devised attributes {*o*_1_, *o*_2_, … *o*_*n*_} and *t* given experts {*d*_1_, *d*_2_, … *d*_*t*_}, let expert’s weight be {*a*_1_, *a*_2_, … *a*_*t*_}, *w* = (*w*_1_, *w*_2_, ⋯, *w*_*n*_) is weight of attributes *o*_*j*_(*j* = 1,2,⋯, *n*), *w*_*j*_ ∈ [0,1], $\sum_{j=1}^{n}w_{j}=1$. *H* is a sort of partially known weight, which has the following forms, for *i* ≠ *j* [42, 43]: Case 1. A weak ranking: *w*_*i*_ ≥ *w*_*j*_; Case 2. A strict ranking: *w*_*i*_ − *w*_*j*_ ≥ *α*_*i*_, *α*_*i*_ > 0; Case 3. A ranking of differences: *w*_*i*_ − *w*_*j*_ ≥ *w*_*k*_ − *w*_*l*_, for *j* ≠ *k* ≠ *l*; Case 4. A ranking with multiples: *w*_*i*_ ≥ *β*_*i*_*w*_*j*_, 0 ≤ *β*_*i*_ ≤ 1; Case 5. An interval form: *α*_*i*_ ≤ *w*_*i*_ ≤ *α*_*i*_ + *ε*_*i*_, 0 ≤ *α*_*i*_ < *α*_*i*_ + *ε*_*i*_ ≤ 1. The steps of 2TLNN-GRA method for MAGDM are devised.

**Step 1**. Build the 2TLNN matrix $R={\left[\phi_{ij}^{t}\right]}_{m\times n},i=1,2,\ldots ,m,j=1,2,\ldots ,n$:

$$\begin{array}{l} \;\;\;\;\;\;\;\;\;\;\begin{array}{cccc} o_{\text{1}} & \;\;o_{\text{2}} & \ldots & o_{n} \end{array}\\ R={\left[\phi_{ij}^{t}\right]}_{m\times n}=\begin{array}{c} \phi_{1}\\ \phi_{2}\\ \vdots \\ \phi_{m} \end{array}\left[\begin{array}{cccc} \phi_{11}^{t} & \phi_{12}^{t} & \ldots & \phi_{1n}^{t}\\ \phi_{21}^{t} & \phi_{22}^{t} & \ldots & \phi_{2n}^{t}\\ \vdots & \vdots & \vdots & \vdots \\ \phi_{m1}^{t} & \phi_{m2}^{t} & \ldots & \phi_{mn}^{t} \end{array}\right] \end{array}$$ (12)

where $\phi_{ij}^{t}=\left\{{\left(s_{t_{ij}},\alpha_{ij}\right)}^{t},{\left(s_{i_{ij}},\beta_{ij}\right)}^{t},{\left(s_{f_{ij}},\chi_{ij}\right)}^{t}\right\}$ is 2TLNNs.

**Step 2**. Obtain average matrix *VR* = [*vϕ*_*ij*_]_*m*×*n*_:

$$\begin{array}{l} \;\;\;\;\;\;\;\begin{array}{cccc} \;\;\;\;\;o_{\text{1}} & \;\;o_{\text{2}} & \;\ldots & \;o_{n} \end{array}\\ VR={\left[v\phi_{ij}\right]}_{m\times n}=\begin{array}{c} \phi_{1}\\ \phi_{2}\\ \vdots \\ \phi_{m} \end{array}\left[\begin{array}{cccc} v\phi_{11} & v\phi_{12} & \ldots & v\phi_{1n}\\ v\phi_{21} & v\phi_{22} & \ldots & v\phi_{2n}\\ \vdots & \vdots & \vdots & \vdots \\ v\phi_{m1} & v\phi_{m2} & \ldots & v\phi_{mn} \end{array}\right] \end{array}$$ (13)

Based on 2TLNNWG operator, the *VR* = [*vϕ*_*ij*_]_*m*×*n*_ is:

$$\begin{array}{l} v\phi_{ij}=\;{\left(\phi_{ij}^{1}\right)}^{a_{1}}⊗{\left(\phi_{ij}^{2}\right)}^{a_{2}}\ldots ⊗{\left(\phi_{ij}^{t}\right)}^{a_{t}}=\overset{t}{\underset{d=1}{⊗}}{\left(\phi_{ij}^{d}\right)}^{a_{d}}\\ =\left\{\begin{array}{l} \Delta \left(M\prod_{d=1}^{t}{\left(\frac{\Delta^{-1}{\left(ls_{t_{ij}},\alpha_{ij}\right)}^{t}}{M}\right)}^{a_{t}}\right),\Delta \left(M\left(1-\prod_{d=1}^{t}{\left(1-\frac{\Delta^{-1}{\left(ls_{i_{ij}},\beta_{ij}\right)}^{t}}{M}\right)}^{a_{t}}\right)\right),\\ \Delta \left(M\left(1-\prod_{d=1}^{t}{\left(1-\frac{\Delta^{-1}{\left(ls_{f_{ij}},\chi_{ij}\right)}^{t}}{M}\right)}^{a_{t}}\right)\right) \end{array}\right\} \end{array}$$ (14)

**Step 3**. Normalize the *VR* = [*vϕ*_*ij*_]_*m*×*n*_ into *NR* = [*nϕ*_*ij*_]_*m*×*n*_.

For benefit attributes:

$$\begin{array}{l} n\phi_{ij}=\left\{\left(ls_{t_{ij}},\alpha_{ij}\right),\left(ls_{i_{ij}},\beta_{ij}\right),\left(ls_{f_{ij}},\chi_{ij}\right)\right\}\\ =\left\{\left(ls_{t_{ij}},\alpha_{ij}\right),\left(ls_{i_{ij}},\beta_{ij}\right),\left(ls_{f_{ij}},\chi_{ij}\right)\right\} \end{array}$$ (15)

For cost attributes:

$$n\phi_{ij}=\left\{\begin{array}{l} \left(ls_{t_{ij}},\alpha_{ij}\right),\\ \left(ls_{i_{ij}},\beta_{ij}\right),\\ \left(ls_{f_{ij}},\chi_{ij}\right) \end{array}\right\}=\left\{\begin{array}{l} \Delta \left(M-\Delta^{-1}\left(ls_{t_{ij}},\alpha_{ij}\right)\right),\\ \Delta \left(M-\Delta^{-1}\left(ls_{i_{ij}},\beta_{ij}\right)\right),\\ \Delta \left(M-\Delta^{-1}\left(ls_{f_{ij}},\chi_{ij}\right)\right) \end{array}\right\}$$ (16)

**Step 4**. Determine the 2TLNN positive ideal solution (2TLNNPIS) and 2TLNN negative ideal solution (2TLNNNIS) through Eqs (17)–(22):

$$2TLNNPIS=\left\{2TLNNPIS_{j},j=1,2,\ldots ,n\right\}.$$ (17)

$$2TLNNNIS=\left\{2TLNNNIS_{j},j=1,2,\ldots ,n\right\}.$$ (18)

$$2TLNNPIS_{j}=\left\{\left(\left(ls_{t_{j}}^{+},\alpha_{j}^{+}\right),\left(ls_{i_{j}}^{+},\beta_{j}^{+}\right),\left(ls_{f_{j}}^{+},\chi_{j}^{+}\right)\right),j=1,2,\ldots ,n\right\}.$$ (19)

$$2TLNNNIS_{j}=\left\{\left(\left(ls_{t_{j}}^{-},\alpha_{j}^{-}\right),\left(ls_{i_{j}}^{-},\beta_{j}^{-}\right),\left(ls_{f_{j}}^{-},\chi_{j}^{-}\right)\right),j=1,2,\ldots ,n\right\}.$$ (20)

$$s\left(\left\{\left(ls_{t_{j}}^{+},\alpha_{j}^{+}\right),\left(ls_{i_{j}}^{+},\beta_{j}^{+}\right),\left(ls_{f_{j}}^{+},\chi_{j}^{+}\right)\right\}\right)=\underset{i}{\text{min}}s\left(\left\{\left(ls_{t_{ij}},\alpha_{ij}\right),\left(ls_{i_{ij}},\beta_{ij}\right),\left(ls_{f_{ij}},\chi_{ij}\right)\right\}\right)$$ (21)

$$s\left(\left\{\left(ls_{t_{j}}^{-},\alpha_{j}^{-}\right),\left(ls_{i_{j}}^{-},\beta_{j}^{-}\right),\left(ls_{f_{j}}^{-},\chi_{j}^{-}\right)\right\}\right)=\underset{i}{\text{min}}s\left(\left\{\left(ls_{t_{ij}},\alpha_{ij}\right),\left(ls_{i_{ij}},\beta_{ij}\right),\left(ls_{f_{ij}},\chi_{ij}\right)\right\}\right)$$ (22)

**Step 5**. Compute the grey rational coefficients (GRC) from the 2TLNNPIS and 2TLNNNIS as:

$$\begin{array}{l} 2TLNNPISGRC\left(\xi_{ij}\right)\\ =\frac{\underset{1\leq i\leq m}{\text{min}}ED\left(N_{ij},2TLNNPIS_{j}\right)+\rho \underset{1\leq i\leq m}{\text{max}}ED\left(N_{ij},2TLNNPIS_{j}\right)}{ED\left(N_{ij},2TLNNPIS_{j}\right)+\rho \underset{1\leq i\leq m}{\text{max}}ED\left(N_{ij},2TLNNPIS_{j}\right)}\\ i=1,2,\cdots ,m,j=1,2,\cdots ,n, \end{array},$$ (23)

$$\begin{array}{l} 2TLNNNISGRC\left(\xi_{ij}\right)\\ =\frac{\underset{1\leq i\leq m}{\text{min}}ED\left(N_{ij},2TLNNNIS_{j}\right)+\rho \underset{1\leq i\leq m}{\text{max}}ED\left(N_{ij},2TLNNNIS_{j}\right)}{ED\left(N_{ij},2TLNNNIS_{j}\right)+\rho \underset{1\leq i\leq m}{\text{max}}ED\left(N_{ij},2TLNNNIS_{j}\right)}\\ i=1,2,\cdots ,m,j=1,2,\cdots ,n, \end{array}$$ (24)

where *ED*(*N*_*ij*_, 2*TLNNPIS*_*j*_) and *ED*(*N*_*ij*_, 2*TLNNPIS*_*j*_) is 2TLNN Euclidean distances.

**Step 6**. Compute the grey relation degree (GRD) of defined alternatives from 2TLNNPIS and 2TLNNNIS:

$$2TLNNPISGRD\left(\xi_{i}\right)=\sum_{j=1}^{n}w_{j}2TLNNPISGRC\left(\xi_{ij}\right),i=1,2,\cdots ,m,$$ (25)

$$2TLNNNISGRD\left(\xi_{i}\right)=\sum_{j=1}^{n}w_{j}2TLNNNISGRC\left(\xi_{ij}\right),i=1,2,\cdots ,m,$$ (26)

The fundamental idea of GRA method is that the optimal alternative is supposed to possess the “largest degree of GRC” from 2TLNNPIS and “smallest degree of GRC” from 2TLNNNIS. Evidently, the larger 2*TLNNPISGRD*(*ξ*_*i*_) along with smaller 2*TLNNNISGRD*(*ξ*_*i*_), the better alternative *ϕ*_*i*_ is. But the attribute weights’ information is incompletely known. So, to derive the *PLPIS*(*ξ*_*i*_), *PLNIS*(*ξ*_*i*_), we can build the multiple objective optimization models (MOOM-1):

$$\left\{\begin{array}{l} \text{max}\;2TLNNPISGRD\left(\xi_{i}\right)=\sum_{j=1}^{n}w_{j}2TLNNPISGRC\left(\xi_{ij}\right)\\ \text{min}\;2TLNNNISGRD\left(\xi_{i}\right)=\sum_{j=1}^{n}w_{j}2TLNNNISGRC\left(\xi_{ij}\right)\\ subject\;to:\;w\in H,i=1,2,\cdots ,m. \end{array}\right.$$

Due to each decision alternative is non-inferior, there is no preference relation for all the decision alternatives. Besides, the multiple objective optimization (MOOM-1) might be fused into the single objective optimization (SOOM-1) with equal weights:

$$\left\{\begin{array}{l} \text{min}\;2TLNNPIS\left(\xi \right)=\sum_{i=1}^{m}w_{j}\left(2TLNNPISGRD\left(\xi_{i}\right)-2TLNNNISGRD\left(\xi_{i}\right)\right)\\ =\sum_{i=1}^{m}\sum_{j=1}^{n}w_{j}\left(2TLNNPISGRD\left(\xi_{ij}\right)-2TLNNNISGRD\left(\xi_{ij}\right)\right)\\ \;=\sum_{i=1}^{m}\sum_{j=1}^{n}w_{j}\left(\begin{array}{l} \frac{\underset{1\leq i\leq m}{\text{min}}ED\left(N_{ij},2TLNNPIS_{j}\right)+\rho \underset{1\leq i\leq m}{\text{max}}ED\left(N_{ij},2TLNNPIS_{j}\right)}{ED\left(N_{ij},2TLNNPIS_{j}\right)+\rho \underset{1\leq i\leq m}{\text{max}}ED\left(N_{ij},2TLNNPIS_{j}\right)}-\\ \frac{\underset{1\leq i\leq m}{\text{min}}ED\left(N_{ij},2TLNNNIS_{j}\right)+\rho \underset{1\leq i\leq m}{\text{max}}ED\left(N_{ij},2TLNNNIS_{j}\right)}{ED\left(N_{ij},2TLNNNIS_{j}\right)+\rho \underset{1\leq i\leq m}{\text{max}}ED\left(N_{ij},2TLNNNIS_{j}\right)} \end{array}\right)\\ subject\;to:\;w\in H \end{array}\right.$$

By solving the (SOOM-1), the solution *w* = (*w*_1_, *w*_2_, ⋯, *w*_*n*_) is regarded as the attributes weight. Then, the 2*TLNNPISGRD*(*ξ*_*i*_) and 2*TLNNNISGRD*(*ξ*_*i*_) is obtained through Eqs (25) and (26).

**Step 7**. Obtain the 2TLNN relative relational degree (2TLNNRRD) from 2TLNNPIS:

$$2TLNNRRD\left(\xi_{i}\right)=\frac{2TLNNNISGRD\left(\xi_{i}\right)}{2TLNNPISGRD\left(\xi_{i}\right)+2TLNNNISGRD\left(\xi_{i}\right)},i=1,2,\ldots ,m,$$ (27)

**Step 8**. According to 2*TLNNRRD*(*ξ*_*i*_). The highest information value of 2*TLNNRRD*(*ξ*_*i*_) is, the optimal alternative is designed.

## 5. The numerical example and comparative analysis

### 5.1. Numerical example

The construction industry is a pillar industry of China’s economy, and plays an important supporting role in my country’s national economy and social development. With the implementation of the "One Belt, One Road" policy, the construction industry will also reach a new stage of development. Of course, opportunities and challenges coexist. How to better combine the characteristics of contemporary enterprise development, achieve higher economic benefits, and then improve international competitiveness is a topic worthy of in-depth study and consideration by Chinese construction enterprises. Under the new situation, construction enterprises should actively carry out reforms, adopt advanced management methods, improve corresponding management systems, and improve management efficiency and social influence. In the process of construction enterprises implementing engineering projects, the choice of material suppliers is very important, and its pros and cons will directly affect the quality, progress and cost of engineering construction. Choosing a suitable building material supplier can, on the one hand, meet the index requirements of all aspects of the project and meet the owner’s need for product excellence, thereby improving customer satisfaction; win. Therefore, it is of great significance to investigate the building materials supplier selection and improve the structure of the entire supply chain. At present, with the changes in the market situation, the requirements of the owners continue to increase, the development environment of construction enterprises has become more diverse, complex and unpredictable, and the competition has become more intense. What used to be simple competition between companies in the same industry has now developed into a complex competition model involving the entire supply chain. With the continuous improvement of customers’ requirements for product quality, after-sales service, corporate image, corporate reputation and other aspects of enterprises, the pressure of enterprises’ survival and competition is also increasing. The development of information technology has also reduced the internal transaction costs of enterprises, which in turn makes the product life cycle is shorter. Therefore, a high-quality supply chain structure is particularly important in the brutal market competition. The typhoon vulnerability assessment of civil engineering structures is a classical MAGDM issues. In this given section, we provide a real numerical example for typhoon vulnerability assessment of civil engineering structures through 2TLNN-GRA method. Assume that five possible civil engineering structures *CES*_*i*_ (*i* = 1,2,3,4,5) to be chosen and four attributes to be assessed these civil engineering structures: ①PQ is the product quality; ②DC is the delivery capacity; ③SL is the service level; ④EP is the enterprise performance. The five possible civil engineering structures *CES*_*i*_ (*i* = 1,2,3,4,5) are to be evaluated by 2TLNNs under the four given attributes by three experts *d*^*t*^ (the expert’s weight is (0.325,0.364,0.311) and known attribute’s weight is *H* = {0.17 ≤ *ω*_1_ ≤ 0.25, 0.16 ≤ *ω*_2_ ≤ 0.25, 0.28 ≤ *ω*_3_ ≤ 0.35, *ω*_3_ − *ω*_4_ ≥ 0.10}.

The 2TLNN-GRA method is used to solve the typhoon vulnerability assessment of civil engineering structures.

**Step 1**. Build the 2TLNN matrix $R={\left[\phi_{ij}^{t}\right]}_{m\times n}$ (See Tables 1–3).

**Table 1:** The 2TLNN information by the first expert.

	PQ	DC
CES_1_	{(ls_3_, 0), (ls_2_, 0), (ls_5_, 0)}	{(ls_1_, 0), (ls_5_, 0), (ls_2_, 0)}
CES_2_	{(ls_2_, 0), (ls_2_, 0), (ls_3_, 0)}	{(ls_2_, 0), (ls_3_, 0), (ls_4_, 0)}
CES_3_	{(ls_3_, 0), (ls_2_, 0), (ls_5_, 0)}	{(ls_2_, 0), (ls_4_, 0), (ls_5_, 0)}
CES_4_	{(ls_5_,0), (ls_2_,0), (ls_3_,0)}	{(ls_5_,0), (ls_2_,0), (ls_3_,0)}
CES_5_	{(ls_4_, 0), (ls_3_, 0), (ls_2_, 0)}	{(ls_5_, 0), (ls_1_, 0), (ls_2_, 0)}
	SL	EP
CES_1_	{(ls_5_, 0), (ls_2_, 0), (ls_3_, 0)}	{(ls_2_, 0), (ls_4_, 0), (ls_3_, 0)}
CES_2_	{(ls_2_, 0), (ls_1_, 0), (ls_5_, 0)}	{(ls_2_, 0), (ls_3_, 0), (ls_4_, 0)}
CES_3_	{(ls_5_, 0), (ls_2_, 0), (ls_1_, 0)}	{(ls_2_, 0), (ls_4_, 0), (ls_3_, 0)}
CES_4_	{(ls_4_, 0), (ls_3_, 0), (ls_1_, 0)}	{(ls_4_,0), (ls_2_,0), (ls_1_,0)}
CES_5_	{(ls_1_, 0), (ls_2_, 0), (ls_4_, 0)}	{(ls_2_, 0), (ls_4_, 0), (ls_5_, 0)}

**Table 2:** The 2TLNN information by the second expert.

	PQ	DC
CES_1_	{(ls_5_, 0), (ls_4_, 0), (ls_4_, 0)}	{(ls_2_, 0), (ls_5_, 0), (ls_4_, 0)}
CES_2_	{(ls_5_, 0), (ls_3_, 0), (ls_4_, 0)}	{(ls_1_, 0), (ls_4_, 0), (ls_3_, 0)}
CES_3_	{(ls_1_, 0), (ls_2_, 0), (ls_4_, 0)}	{(ls_4_, 0), (ls_2_, 0), (ls_3_, 0)}
CES_4_	{(ls_2_, 0), (ls_1_, 0), (ls_4_, 0)}	{(ls_1_, 0), (ls_3_, 0), (ls_5_, 0)}
CES_5_	{(ls_4_, 0), (ls_1_, 0), (ls_2_, 0)}	{(ls_5_, 0), (ls_2_, 0), (ls_1_, 0)}
	SL	EP
CES_1_	{(ls_3_, 0), (ls_2_, 0), (ls_5_, 0)}	{(ls_1_, 0), (ls_3_, 0), (ls_4_, 0)}
CES_2_	{(ls_2_, 0), (ls_4_, 0), (ls_1_, 0)}	{(ls_3_, 0), (ls_5_, 0), (ls_2_, 0)}
CES_3_	{(ls_2_, 0), (ls_3_, 0), (ls_4_, 0)}	{(ls_4_, 0), (ls_2_, 0), (ls_1_, 0)}
CES_4_	{(ls_3_, 0), (ls_4_, 0), (ls_2_, 0)}	{(ls_3_, 0), (ls_5_, 0), (ls_2_, 0)}
CES_5_	{(ls_4_, 0), (ls_1_, 0), (ls_2_, 0)}	{(ls_5_, 0), (ls_3_, 0), (ls_2_, 0)}

**Table 3:** The 2TLNN information by the third expert.

	PQ	DC
CES_1_	{(ls_2_, 0), (ls_3_, 0), (ls_1_, 0)}	{(ls_4_, 0), (ls_2_, 0), (ls_3_, 0)}
CES_2_	{(ls_4_, 0), (ls_5_, 0), (ls_4_, 0)}	{(ls_3_, 0), (ls_4_, 0), (ls_3_, 0)}
CES_3_	{(ls_1_, 0), (ls_1_, 0), (ls_4_, 0)}	{(ls_2_, 0), (ls_1_, 0), (ls_5_, 0)}
CES_4_	{(ls_2_, 0), (ls_3_, 0), (ls_4_, 0)}	{(ls_4_, 0), (ls_3_, 0), (ls_1_, 0)}
CES_5_	{(ls_5_, 0), (ls_1_, 0), (ls_1_, 0)}	{(ls_5_, 0), (ls_2_, 0), (ls_1_, 0)}
	SL	EP
CES_1_	{(ls_4_, 0), (ls_2_, 0), (ls_5_, 0)}	{(ls_3_, 0), (ls_2_, 0), (ls_1_, 0)}
CES_2_	{(ls_2_, 0), (ls_4_, 0), (ls_1_, 0)}	{(ls_4_, 0), (ls_5_, 0), (ls_2_, 0)}
CES_3_	{(ls_3_, 0), (ls_1_, 0), (ls_5_, 0)}	{(ls_2_, 0), (ls_2_, 0), (ls_4_, 0)}
CES_4_	{(ls_2_,0), (ls_4_, 0), (ls_3_, 0)}	{(ls_1_, 0), (ls_3_, 0), (ls_2_, 0)}
CES_5_	{(ls_4_, 0), (ls_1_, 0), (ls_2_, 0)}	{(ls_5_, 0), (ls_3_, 0), (ls_4_, 0)}

**Step 2**. Normalize the $R={\left[\varphi_{ij}^{r}\right]}_{5\times 4}$ to $R^{\prime }={\left[{\varphi^{\prime }}_{ij}^{r}\right]}_{5\times 4}$, for all the given attributes are benefit, the normalization is not really needed.

**Step 3**. According to $R={\left[\varphi_{ij}^{r}\right]}_{m\times n}$ and expert’s weight (0.325,0.364,0.311). The average matrix is presented in Table 4 based on 2TLNNWG operator.

**Table 4:** The average matrix with 2TLNNWG operator.

	PQ	DC
CES_1_	{(ls_2_, 0.219), (ls_3_, -0.347), (ls_3_, -0.176)}	{(ls_1_, 0.194), (ls_2_, 0.291), (ls_2_, 0.497)}
CES_2_	{(ls_5_, -0.433), (ls_4_, 0.167), (ls_4_, -0.213)}	{(ls_5_, 0.034), (ls_2_, 0.052), (ls_1_, 0.286)}
CES_3_	{(ls_3_, 0.169), (ls_4_, 0.498), (ls_2_, 0.462)}	{(ls_2_, 0.421), (ls_3_, 0.038), (ls_2_, 0.263)}
CES_4_	{(ls_3_, 0.431), (ls_2_, 0.343), (ls_3_, 0.157)}	{(ls_3_, -0.345), (ls_3_, 0.212), (ls_4_, -0.325)}
CES_5_	{(ls_2_, 0.176), (ls_2_, -0.362), (ls_3_, -0.216)}	{(ls_3_, 0.076), (ls_2_, -0.221), (ls_3_, -0.298)}
	SL	EP
CES_1_	{(ls_2_, 0.254), (ls_3_, -0.442), (ls_4_, 0.043)}	{(ls_2_, 0.225), (ls_3_, 0.189), (ls_1_, 0.162)}
CES_2_	{(ls_2_, 0.021), (ls_4_, 0.287), (ls_1_, -0.256)}	{(ls_5_, -0.159), (ls_2_, 0.234), (ls_3_, -0.292)}
CES_3_	{(ls_3_, -0.032), (ls_2_, 0.015), (ls_5_, 0.169)}	{(ls_3_, -0.196), (ls_2_, 0.147), (ls_2_, -0.052)}
CES_4_	{(ls_2_, 0.212), (ls_4_, -0.465), (ls_1_, 0.261)}	{(ls_3_, -0.345), (ls_3_, 0.212), (ls_4_, -0.325)}
CES_5_	{(ls_3_, 0.312), (ls_3_, -0.236), (ls_5_, -0.479)}	{(ls_3_, 0.076), (ls_2_, -0.221), (ls_3_, -0.298)}

**Step 4**. Determine the 2TLNNPIS and 2TLNNNIS (See Table 5).

**Table 5:** The 2TLNNPIS and 2TLNNNIS.

	PQ	DC
2TLNNPIS	{(ls_5_, -0.433), (ls_4_, 0.167), (ls_4_, -0.213)}	{(ls_5_, 0.034), (ls_2_, 0.052), (ls_1_, 0.286)}
2TLNNNIS	{(ls_2_, 0.176), (ls_2_, -0.362), (ls_3_, -0.216)}	{(ls_3_, 0.076), (ls_2_, -0.221), (ls_3_, -0.298)}
	SL	EP
2TLNNPIS	{(ls_3_, -0.032), (ls_2_, 0.015), (ls_5_, 0.169)}	{(ls_5_, -0.159), (ls_2_, 0.234), (ls_3_, -0.292)}
2TLNNNIS	{(ls_2_, 0.254), (ls_3_, -0.442), (ls_4_, 0.043)}	{(ls_2_, 0.225), (ls_3_, 0.189), (ls_1_, 0.162)}

**Step 5**. Compute the 2*TLNNNISGRC*(*ξ*_*ij*_) and 2*TLNNNISGRC*(*ξ*_*ij*_) (See Tables 6 and 7).

**Table 6:** The 2*TLNNNISGRC*(*ξ*_*ij*_).

Alternatives	PQ	DC	SL	EP
CES_1_	0.7824	1.0000	0.4332	0.5094
CES_2_	0.6442	0.5342	0.5174	0.5942
CES_3_	0.8048	0.7824	1.0000	1.0000
CES_4_	0.6180	0.5942	0.5342	0.5830
CES_5_	1.0000	0.5342	0.5174	0.6180

**Table 7:** The 2*TLNNNISGRC*(*ξ*_*ij*_).

Alternatives	PQ	DC	SL	EP
CES_1_	0.8415	1.0000	0.7410	0.7788
CES_2_	0.5698	1.0000	1.0000	0.7854
CES_3_	0.7655	0.6902	1.0000	1.0000
CES_4_	1.0000	0.8415	1.0386	0.6723
CES_5_	1.0000	0.7788	0.8082	0.8012

**Step 6**. The model (SOOM-1) is utilized to set up the single-objective programming model:

$$\left\{\begin{array}{l} \text{min}\;d(w)=-0.1437w_{1}-0.05381w_{2}+0.0359w_{3}-0.1435w_{4}\\ subject\;to\;w\in H \end{array}\right.$$

The weight of attributes is obtained: *w* = (0.2500, 0.1700, 0.3500, 0.2300)^*T*^.

**Step 7**. Compute the 2*TLNNPISGRD*(*ξ*_*i*_) and 2*TLNNNISGRD*(*ξ*_*i*_) (See Table 8):

**Table 8:** The 2*TLNNPISGRD*(*ξ*_*i*_) and 2*TLNNNISGRD*(*ξ*_*i*_).

Alternatives	2*TLNNPISGRD*(*ξ*_*i*_)	2*TLNNNISGRD*(*ξ*_*i*_)
CES_1_	0.4351	0.4197
CES_2_	0.5535	0.6859
CES_3_	0.7685	0.4027
CES_4_	0.4995	0.302
CES_5_	0.5192	0.3841

**Step 8**. Compute each alternative’s 2*TLNNRRD*(*ξ*_*i*_) (See Table 9).

**Table 9:** The alternative’s 2*TLNNRRD*(*ξ*_*i*_) from 2TLNNNIS.

Alternatives	2*TLNNRRD*(*ξ*_*i*_)	Order
CES_1_	0.6184	2
CES_2_	0.6992	1
CES_3_	0.4301	5
CES_4_	0.4481	4
CES_5_	0.5259	3

**Step 9**. According to 2*TLNNRRD*(*ξ*_*i*_), the order is *CES*_2_ > *CES*_1_ > *CES*_5_ > *CES*_4_ > *CES*_3_ and *CES*_2_ is the best one.

### 5.2 Compare 2TLNN-GRA with some 2TLNNs operators

In such section, the 2TLNN-GRA method is compared with 2TLNWHM and 2TLNWDHM operator [13]. The fused information values through two operators are given in Table 10.

**Table 10:** The fused information values through two operators.

	2TLNWHM operator	2TLNWDHM operator
CES_1_	{(ls_4_, -0.476), (ls_3_, 0.245), (ls_4_, 0.476)}	{(ls_3_, 0.348), (ls_3_, 0.210), (ls_3_, -0.304)}
CES_2_	{(ls_3_, 0.113), (ls_3_, -0.142), (ls_4_, -0.103)}	{(ls_2_, -0.129), (ls_2_, -0.107), (ls_3_, -0.125)}
CES_3_	{(ls_2_, 0.085), (ls_2_, 0.054), (ls_4_, -0.085)}	{(ls_2_, 0.421), (ls_2_, 0.145), (ls_3_, -0.201)}
CES_4_	{(ls_3_, -0.034), (ls_4_, -0.206), (ls_2_, 0.027)}	{(ls_4_, -0.253), (ls_2_, -0.164), (ls_2_, 0.253)}
CES_5_	{(ls_2_, 0.343), (ls_4_, -0.017), (ls_3_, -0.393)}	{(ls_2_, 0133), (ls_4_, 0.067), (ls_4_, -0.149)}

According to score of 2TLNNs, the score for alternative is listed in Table 11.

**Table 11:** Scores of given alternatives.

Alternatives	2TLNWHM operator	2TLNWDHM operator
S(CES_1_)	0.8609	0.5579
S(CES_2_)	0.9793	0.7241
S(CES_3_)	0.8943	0.6409
S(CES_4_)	0.7853	0.5374
S(CES_5_)	0.875	0.6223

The order by 2TLNNs operators is obtained in Table 12.

**Table 12:** Order through 2TLNNs operators.

	order
2TLNWHM operator [13]	*CES*_2_ > *CES*_3_ > *CES*_5_ > *CES*_1_ > *CES*_4_
2TLNWDHM operator [13]	*CES*_2_ > *CES*_3_ > *CES*_5_ > *CES*_1_ > *CES*_4_
2TLNN-GRA method	*CES*_2_ > *CES*_1_ > *CES*_5_ > *CES*_4_ > *CES*_3_

Comparing the results of the 2TLNN-GRA method with 2TLNWHM & 2TLNWDHM fused operators, the obtained results are slightly different and the chosen best alternative is same. However, the 2TLNN-GRA has the precious characteristics: (1) the basic idea of 2TLNN-GRA is to judge whether the relationship between the sequences is close according to the similarity of the shape of the sequence curves; if the curves between the sequences are closer, the greater the degree of correlation between the corresponding sequences, and vice versa; (2) 2TLNN-GRA is based on the development trend, so there are no too many requirements for the size of the sample, nor does it need a typical distribution law, and the amount of calculation is relatively small, the results will be more consistent with the qualitative analysis results. Therefore, the GRA is a relatively simple and reliable analysis method in system analysis.

## 6. Conclusion

In recent years, some researchers in the field of civil engineering disaster science have gone deep into the typhoon-stricken areas to investigate the typhoon damage of civil engineering structures, and analyze and summarize the experience of structural typhoon disasters based on the damage degree and damage characteristics of various engineering structures. These experiences truly reflect the impact of typhoons on engineering structures, and comprehensively reveal the actual wind resistance performance of various engineering structures. It can be seen that using the existing structural typhoon disaster data to evaluate the wind resistance performance of various existing engineering structures is an important aspect of wind engineering research. In the past five years, the typhoon disaster of low-rise buildings in the southeast coastal villages and towns of my country has been particularly serious, which has seriously affected the goal of building a harmonious society for the coordinated development of urban and rural areas in my country. Therefore, we must quickly strengthen the regional typhoon disaster investigation of low-rise buildings to obtain more abundant structural typhoon disaster data, and to achieve structural typhoon vulnerability assessment and loss estimation. Therefore, it is very important to use scientific and effective methods for typhoon vulnerability assessment of civil engineering structures. The typhoon vulnerability assessment of civil engineering structures is the MAGDM. In this paper, we build the 2TLNN-GRA method for MAGDM based on the traditional GRA method. Finally, a numerical example for typhoon vulnerability assessment of civil engineering structures has been given to illustrate the 2TLNN-GRA method. Thus, the main research contribution of this study is: (1) the 2TLNN-GRA method is used to deal with the MAGDM problems under 2TLNNs with incomplete weight information; (2) an empirical example for typhoon vulnerability assessment of civil engineering structures has been given. (3) some comparative algorithms are given to show the rationality of 2TLNN-GRA method. In the future, the 2TLNN-GRA method could be applied to the risk analysis issues, selection issues, other MAGDM issues and many other uncertain environments.

According to the current research status in this field and its own research progress, research and exploration of decision-making and evaluation methods will be continued in the following aspects in the future. (1) Consensus and consistency improvement may conflict with each other in group decision-making [44–50], so it is a decision and evaluation worthy of research to construct a new consistency and consensus improvement model with the help of the two-level programming model and combine the genetic algorithm to solve it method question [51, 52]. (2) This paper mainly studies the small-scale group decision-making problem in the 2TLNNs environment. Extending the GDM method of large groups and social networks to the 2TLNNs environment is a problem worthy of further research [53, 54]. (3) The operator proposed in this paper is improved to consider the expression of decision evaluation information based on language preference relationship, such as group decision method based on probabilistic linguistic decision information [55, 56] and probabilistic uncertain linguistic decision information [57, 58], which is also a topic worthy of future research.
